# Research on Cardiorespiratory Endurance Test and Training Method Based on Structural Equation Model

This article has been retracted.

**DOI:** 10.1155/2022/7604856

**Published:** 2022-03-07

**Authors:** Jianmin Wang

**Affiliations:** Department of Physical Education and Teaching, Huaiyin Institute of Technology, Huai'an, Jiangsu 223003, China

## Abstract

In order to study the cardiorespiratory endurance test and training method under the structural equation model, a structural equation model built in conjunction with ANOS7.0 is proposed. This method uses confirmatory factor analysis and analyzes the influencing factors of motor skills. Studies indicate that df = 173 > 0 of the structural equation model, to over-identify the model, the absolute value of the standardized coefficient value is 0.257 to 0.758, less than 0.95, and there is no value with a large estimated standard deviation. The model did not violate the estimation phenomenon. Among the factors affecting motor skills, cardiopulmonary function, and muscle endurance, the weight of the back muscles is less than 0.4, the power of coordination and explosive power of lower limbs is greater than 0.6, and limb muscle strength, body mass, and the stretch and flexibility of the muscles have a greater weight on basketball skills than 0.5. The structural equation model is an over-recognition model. The absolute value of the standardized coefficient value does not have a value with an excessively large standard deviation estimate, and the model does not violate the estimate.

## 1. Introduction

Cardiopulmonary function refers to breathing through the lungs from the circulatory system, and heart activity promotes blood circulation to deliver oxygen and nutrients to the body. Cardiopulmonary endurance represents the body's ability to continue physical activity, *t* reflects the cardiopulmonary function of the human body under a certain exercise intensity. It is considered to be one of the most important indicators in the healthy physical fitness evaluation index system [1]. Modern medical research certificate, if the level of cardiorespiratory endurance is low, the risk of suffering from cardiovascular diseases is significantly increased. Improving cardiorespiratory endurance level can not only improve cardiopulmonary adaptability, enhance physical fitness, and improve exercise efficiency, it can also reduce cardiovascular diseases caused by poor lifestyles, the incidence of metabolic diseases and other diseases, and improve people's quality of life [2]. Students who master certain sports skills are more likely to obtain the emotional satisfaction brought about by sports. Students mastering certain motor skills can not only enhance their physical fitness, but also help to develop exercise habits [3]. The study found that the differences in individual sports skills of students are manifested in two aspects: physical fitness and motor skill level. Therefore, studying the relationship between physical fitness and motor skills helps to narrow the individual differences between college students and enables college students to master a sport skill as soon as possible. It is of positive significance to improve the overall physical quality of college students. In summary, how to enable college students to quickly master a sports skill is especially crucial to improve the physical quality of college students. Basketball is an important part of the physical education curriculum in ordinary colleges and universities. Research on how to quickly improve the basketball skills of college students has a demonstrative effect on the development of college students' sports skills [4]. However, this research hopes to study the impact of college students' physical fitness on basketball skills through structural equation modeling. On the basis of previous studies, the aim is to find out how to quickly improve the basketball level of college students by improving their physical fitness, experience the fun of basketball, develop exercise habits, and then improve the overall physical quality of college students [5]. Xue et al. used structural equation models to analyze psychological factors, the mechanism by which school factors and family factors have an effect on exercise behavior [6]. Steinhard et al. used structural equations to construct a verification model to study the influence of physical health beliefs on college students' physical exercise habits [7]. Akilina et al. used structural equation model analysis to analyze the psychological and environmental mechanisms that affect physical exercise behavior [8]. Chen et al. studied the identifiability and estimation function of the causal model when selection bias appears, learned the identifiability between two variables when the selection bias occurs, and the identifiability of the model and the result-dependent choice when the causal direction is given, and put forward the evaluation model for causal inference when there is selection bias. Measurement errors are also very likely to occur during the data acquisition process. Measurement errors in the values of observed variables will greatly change the results of causal discovery methods. So it has also attracted more attention [9].

Based on previous studies, this research uses structural equation modeling to study the impact of college students' physical fitness on basketball skills. The aim is to find out how to quickly improve the basketball level of college students by improving their physical fitness, experience the fun of basketball, develop exercise habits, and then improve the overall physical quality of college students [10].

## 2. Structural Equation Model and Cardiopulmonary Endurance Test Training Method

A graph *G* contains a set of vertices (or nodes) *V* and a set of edges *E* connecting these vertices. The vertices in the graph correspond to variables. The edge is expressed as a certain relationship existing in the pair of variables. The interpretation will vary with the application. Two variables connected by an edge are called adjacent variables. Each edge in the figure can be directional (marked with a single arrow on the edge) or undirected. In some cases, we also use the “two-way” edge to indicate the presence of unobserved confounding factors. It is represented by an arc-shaped dashed arc with two arrows (as shown in Figure 1(a)). If all edges are oriented (as shown in Figure 1(b)), it is called a directed graph. If we remove the arrows on all sides, the resulting unoriented image is called the skeleton of the image *G* (skeleton). Directed graphs may contain directional cycles (such as *X* ⟶ *Y*, *Y* ⟶ *X*) to represent mutual causality or feedback processes, but there can be no self-loops (such as *X* ⟶ *X*). An oriented and acyclic graph is called a directed acyclic graph (DAG), most discussions about causality are based on DAG. A causal graph represented by a directed acyclic graph represents the causal variables in the causal relationship, such as outcome variables, noise variables, and confusion factors, and the mutual causal relationship between variables. The intuitive understanding of causal analysis is of great significance [11].

A structural equation model is a framework for multivariate analysis. It contains variable sets and equation sets.

(1) $$\begin{array}{c} x_{i}=f_{i}\left(pa_{i},u_{i}\right),\;i=1,\ldots ,n. \end{array}$$

Among *pa*_*i*_, stands for *x*_*i*_, a set of direct causes of variables, *u*_*i*_ represents noise or errors caused by some factors. The structural equation model is different from ordinary algebraic equations in that it not only expresses the equality relationship between the two sides of the equation, but it also represents how the variable value on the left side of the equation is generated by the causal mechanism of the variable on the right side. But when the observation data of two variables are given, it is impossible to identify the direction of cause and effect only through the structural equation model. In the nonlinear additive noise model, it is assumed that the observation data are generated in the following way: for each observable variable *x*_*t*_ associated with vertex *i* in the directed acyclic graph *G*, its value is the function of its parent node in graph *G* plus independent noise *u*_*i*_, generated, as follows:

(2) $$\begin{array}{c} x_{i}=f_{i}\left(xpa_{\left(i\right)}\right)+n_{i}, \end{array}$$

where Guan is any function, and it may be different for each *i*; *xpa*_(*i*)_ is a vector containing *x*_*j*_, it has an edge from *j* to *i* in graph *G*; noise variable *n*_*i*_, it can be any probability distribution *p*_*i*_(*n*_*i*_); and the noise variables are independent of each other, namely, *p*_*n*_(*n*)=∏*p*_*ni*_(*ni*), where *n* represents the vector containing the noise variable *n*_*i*_. Given the data vector, the goal of causal discovery is to infer more information about the data generation mechanism. Through the reasoning in the paper, there are the following theorems for the identifiability of the ANM model:

(3) $$\begin{array}{c} p\left(x,y\right)=p_{n}\left(y-f\left(x\right)\right)p_{x}\left(x\right), \end{array}$$

where *p*_*n*_ and *p*_*x*_ are probability distributions, if there is a reverse model of the same form, it is as follows:

(4) $$\begin{array}{c} p\left(x,y\right)=p_{\tilde{n}}\left(x-g\left(y\right)\right)p_{y}\left(y\right). \end{array}$$

From the abovementioned theorem, we can see that given the observation data, if the data can meet ANM's forward model and reverse model at the same time, the triple (*f*, *p*_*x*_, *p*_*n*_) must satisfy formula (4); that is, in most cases, the forward model and the reverse model cannot be established at the same time. It also shows that the ANM model can distinguish the direction of cause and effect in most cases. The algorithm flow of the ANM model to identify the causal direction is as follows:

1. Check whether *x* and *Y* are statistically independent, if they are not, perform the following operations:
2. Detection model *y*=*f*(*x*)+*n*, whether it meets the data, that is, to perform nonlinear regression to get the estimated $\hat{f}$ of the function *f*, calculate the corresponding residual $\hat{n}=y-\hat{f}\left(x\right)$, and then check whether $\hat{n}$ is independent of *x*
3. If it is not independent, it means that the model is wrong, then check whether the reverse model *x*=*g*(*y*)+*n* conforms to the data

Among these, the choice of nonlinear regression methods and specific independence tests is not restricted. Through the abovementioned algorithm flow, the following situations may occur: first, if *x* and *Y* are statistically independent, we can infer that there is no causal relationship between these two variables, then further analysis is unnecessary. On the other hand, if they are related but the models in both directions are consistent, we can conclude that any model may be correct, but we cannot infer its conclusion from the data. The more positive result is that, when we can reject the model in one of the directions and accept another direction, we can infer that the accepted direction is the correct causal direction. Finally, there may be models in both directions that are inconsistent with the data. In this case, we can conclude that the generation mechanism is more complicated, this cannot be described using the ANM model.

### 2.1. Cardiorespiratory Endurance Test Method Based on Treadmill

The treadmill exercise test is a common cardiorespiratory endurance test method. Traditional treadmill exercise experiments need to be equipped with blood pressure monitoring, ECG detection, breathing gas monitoring, blood oxygen saturation detection, and other equipment. Based on this test system, many indicators and evaluation systems can be obtained from it; however, the process of this test method is complicated, the equipment is expensive and cannot be widely used. In this chapter, a treadmill is selected as the basic exercise equipment, and expensive gas detection and other equipment are abandoned. Based on treadmills and heart rate belts, three cardiopulmonary endurance test methods are designed and implemented; they are the two-level load test, the three-level load test, and the step-by-step load test. The direct test method is taken as a comparative test, and the effectiveness and operability of various indirect test methods are analyzed.

Comprehensive domestic and foreign exercise physiologists on heart rate, exercise intensity, and the study of the relationship between the three oxygen uptakes has led to the conclusion that there is a linear correlation between exercise intensity and heart rate within a certain range. Therefore, a lower exercise intensity can be selected, record exercise intensity separately (FC_1_, FC_2_) and the subject's exercise heart rate (HR_1_, HR_2_) at this intensity is based on the maximum heart rate (HR_max_), then calculate the maximum exercise intensity FC_max_ that the subject can withstand according to the linear relationship. This method of inferring the maximum oxygen uptake through the heart rate and oxygen uptake at two lower exercise intensities is a two-level load indirect test method based on the treadmill exercise protocol. Calculated as follows:

(5) $$\begin{array}{c} \frac{{\text{FC}}_{\max}-{\text{FC}}_{2}}{{\text{HR}}_{\max}-{\text{HR}}_{2}}=\frac{{\text{FC}}_{2}-{\text{FC}}_{1}}{{\text{HR}}_{2}-{\text{HR}}_{1}}. \end{array}$$

## 3. Experimental Analysis

This section selects different two-level loads according to different genders and age groups as the exercise intensity of the two-level load test (Table 1). The treadmill at each stage sets the slope and speed according to the exercise intensity. The analytical method of exercise intensity in the treadmill is introduced in the following chapters. Heart rate is monitored in real time while exercising. According to the exercise intensity and the heart rate of the two phases, find the linear relationship between the subject's intensity and heart rate, and based on the predicted maximum heart rate, the maximum exercise intensity that the subject can withstand is obtained. The direct test method of the exercise protocol as a comparative test is taken. Through data analysis, the effectiveness of the two-level load test method is analyzed.

According to the survey results, in order to allow most healthy people to withstand the maximum exercise intensity in this test method, the intensity of the second stage in the secondary load test method must be set no higher than the intensity of the grade. In addition, in order to reduce the influence of heart rate fluctuations on the test data, try to make the two-stage exercise intensity span as large as possible. Generally, the intensity of the first stage is selected not to be higher than the running limit of the corresponding crowd.

### 3.1. Test Method

Male and female volunteers of all ages as test subjects are selected. In each age group, there are 12 males and females. The subject cannot participate in strenuous exercise hours before the start of the test; they should not overeat; make sure the body is in good condition before the test; not suffering from diseases that affect cardiopulmonary function (such as colds) or diseases that affect normal running (such as fractures); and the tester should wear loose clothing that is convenient for exercise. Before the exercise test, set up files for the subjects in the treadmill software and the equipment software, and fill in basic information such as height, weight, and age accurately. All subjects must read the informed consent form carefully, know the precautions for testing, hazard, and accident handling plan during the test, and perform according to the recommendations of sports instructors and medical staff. Finally, a written informed consent agreement was signed. The subject wears a heart rate belt before the test, does minutes of free exercise on the treadmill, adapts to the rhythm of the treadmill, then rests for a minute, and starts the test when the heart rate is close to the resting state. The subject first exercised for a minute at low intensity. Then, the average of the heart rate in seconds before the end of the test is taken to represent the phase heart rate of the subject under low intensity. Then, they rested for a minute before the second level test, in order to avoid the mutual influence of heart rate between the two levels of load, and finally did high-intensity load exercise for 3 minutes. Similarly, the average value of the heart rate 20 seconds before the end of the test is taken to represent the phase heart rate of the subject under high intensity. Record the exercise intensity and phase heart rate under two levels of load, respectively, get the linear relationship between exercise intensity and heart rate, substitute the maximum heart rate predicted based on age into the linear relationship, find the maximum exercise intensity that the subject can withstand, and this intensity represents the subject's maximum exercise capacity. Play soothing music during a break in the middle of the stage. It is convenient for the subjects to relax. Voice prompts to the subject before the treadmill accelerates or decelerates. During the test, the heart rate curve is displayed in real time. HRInput represents the heart rate value sampled in real time, HRShow represents the heart rate after a sliding average, and the intersection of the red line and the time axis represents the starting point and ending point of each stage.

### 3.2. Result Analysis

The test results of all subjects are integrated, as shown in Figure 2. The horizontal axis represents the maximum exercise intensity obtained by the secondary load test method (FC_max_), the unit is MET; the vertical axis represents the maximum oxygen uptake obtained by the VO2000 test method (VO_2max_), the unit is ml/kg/min; and each dot represents a test subject. A straight line fitting across the origin is chosen. According to the fitting results, it can be seen that two test methods are tested. The results are basically the same, straight line fitting has a significant correlation (*R*_2_=0.63), among VO_2max_=3.4433^*∗*^*F*_*c*max_.

The results of the two-level load test method based on the Bruce treadmill protocol are in good agreement with the results of the VO2000 direct test method. The secondary load test method can basically replace the VO2000 direct test method. In practical applications, the secondary load test method can also be regarded as a simple and effective cardiopulmonary endurance test method.

## 4. Conclusion

The structural equation model is an over-recognition model. The absolute value of the standardized coefficient value does not have a value with an excessively large standard deviation estimate. The model does not violate the estimation phenomenon. The development of exercise guidance programs is inseparable from the development of exercise rehabilitation therapy and motor function assessment. Performance assessment and physical fitness tests are the basis for the execution and implementation of the exercise instruction program. Two types of cardiopulmonary endurance test methods are proposed in combination with health examination equipment and treadmills, and the validity and accuracy of these test methods are verified through experiments. According to the results of a treadmill-based cardiorespiratory endurance test, a scientific fitness guidance program is generated. Certain results have been achieved in the previous studies on cardiopulmonary endurance testing methods and training guidance; however, due to time and conditions, there are still some areas to be improved and perfected.

## Figures and Tables

**Figure 1:** Directed acyclic graph. (a) The graph contains one-way and two-way edges, (b) directed acyclic graphs (DAG) with the same skeleton.

**Figure 2:** Analysis of secondary load test results.

**Table 1:** The exercise intensity, corresponding speed, and slope of the two-level load adjusted according to age and gender.

Age		15–39		40–49		50–59	
		MET	V + A	MET	V + A	MET	V + A
First load	Male	6	5.5, 5	6	5.5, 5	4	4.1, 3
	Female	5	4.9, 4	5	4.4, 5	4	4.1, 3

Second load	Male	8	8.3, 3	9	7.5, 3	7	6.3, 0
	Female	10	7.0, 1	8	7.0, 1	6	5.5, 5

## Data Availability

The data used to support the findings of this study are available from the corresponding author upon request.
